RETRACTED

# Analysis of the Effect of Classroom Reform of English Literature on the Theme of Environmental Protection in Universities Based on Artificial Intelligence Technology

**DOI:** 10.1155/2022/2178579

**Published:** 2022-09-09

**Authors:** Xuefeng Li

**Affiliations:** Sanquan College of Xinxiang Medical University, Xinxiang, Henan 453003, China

## Abstract

Under the current theme of environmental protection, the effect of English literature classroom teaching reform cannot be analyzed qualitatively. Based on BP neural network, we present an analytical model of the impact of College English Literature Classroom Teaching Reform on environmental protection based on artificial intelligence technology. We analyze the teaching reform of English literature classrooms with the theme of environmental protection under artificial intelligence technology and explore the concept of “intelligent education” and the construction path of university English ecological teaching mode. Based on the in-depth excavation of teaching information, this paper analyzes the impact of college English literature classroom reform on the theme of environmental protection. Combined with BP neural network, a scientific analytic hierarchy process index system model is established, and the weight relationship of various reform influencing factors is given relatively objectively. The scores of the model based on the BP neural network under the six effect analysis indicators of teaching attitude, teaching tools, reform plan, reform teaching content, classroom organization, and reform rationality are 90.97, 86.3, 80.4, 95.7, 84.8, and 87.4, respectively. The results show that this model has a good ability for analysis and evaluation, which also provides some new ideas and entry points for the reform of the current English classroom teaching model. This study has a certain contribution to the breakthrough of college English teaching goals.

## 1. Introduction

Artificial intelligence (AI) is considered to be the most disruptive technology so far [1], and it is accelerating its landing and profoundly changing the world and human production and lifestyle [2]. The deep integration and innovation of AI in various fields are disrupting our lives and changing the face of the world [3]. AI has been closely related to education since its birth, and the changes to education will be comprehensive.

The natural environment we live in is the collective wealth given by nature to everyone. Therefore, protecting the environment and maintaining ecological balance has become a consensus that everyone should have. The goal of quality education in China points out that natural environment education should permeate all disciplines. English is the main subject of everyone's education, and it is also a part of the teaching system. Reading is a key way to master language knowledge, acquire language information, and improve language use, and the English literature classroom occupies a key position in the English language learning loop in colleges and universities [4]. In College English teaching, we should carry out literature courses with the theme of natural environment protection and integrate environmental education with artificial intelligence technology into teaching. This will not only help to cultivate students' English reading ability but also help students to pay attention to and protect the natural environment. Core literacy training is one of several critical problems in China's education innovation. Front-line English teachers should actively respond to the needs of the times, profoundly grasp the concept of English core literacy teaching, take effective measures to realize the transformation of high school English teaching from language usability enhancement to subject core literacy training, and emphasize the standardization and cultivation of students' thinking quality and cultural character while focusing on the development of student's learning ability and language ability.

RETRACTED

In today's information age, where an era dominated by science and technology, the progress of AI technology has greatly promoted the innovation and progress of English classroom students' learning methods and English learning concepts. Literature [5] has summarized some English teaching modes combined with artificial intelligence technology, showed a cloud computing artificial intelligence model in the article, discussed the relevant characteristics of the intelligent classroom from the perspective of cloud computing, and reformed the interactive teaching mode to a certain extent. This also provides some new ideas and methods for the follow-up classroom education reform so that we can consider the direction of higher education reform from different perspectives such as big data, cloud computing, and AI. Literature [6] has combined AI to advance teaching reform research, collect data using query analysis, and analyze them given distributed technology and new processes. Literature [7] has taken AI combined with cloud computing technology as the research point, deeply analyzes and studies the role of cloud computing and big data technology in college English classroom teaching reform, and then takes cloud computing and big data as tools to deeply analyze the current situation of college English teaching reform. This model takes educational informatization as the research background, integrates the translation meaning of artificial intelligence technology into classroom teaching, and expounds on the transformation significance of artificial intelligence at the teaching level through practice and theoretical basis. Under the above circumstances, the research path of this paper is established. Among them, the ultimate translational value gained from the integration of AI with teaching is the focus of the research reviewed in this literature. Literature [8] has proposed an implementation scheme for college English auxiliary teaching systems of college based on AI technology. Based on artificial intelligence and College English teaching, some improvements have been made in some aspects of the English teaching system to make the current English teaching system more humanized and more suitable for Contemporary English teaching.

RETRACTED

Starting from the situation of AI technology and traditional English teaching, we have deeply discussed the application of AI technology in English Teaching to improve the quality and effectiveness of English teaching. Literature [9] has used a dataset of 6.6 million entries containing 3.25 million favorable and unfavorable English texts. The model uses the normalization method to preprocess the dataset to eliminate impact noise. Based on the variable automatic encoder (VAE) [10], the relevant discriminant features are extracted, and then the random forest algorithm (RF) is used as the classifier to classify the discriminant features, to obtain accurate performance. The performance of the protocol is measured by the transmission rate, active nodes, energy consumption, and a certain number of transmission packets. Literature [11] has designed a virtual corpus-assisted intelligent English teaching model through AI technology. Part of the reading blocks in English from previous universities is text-centered and text-based. The literature adopts the DDL (data definition language) model such that teachers can break through the limitations of textbooks when they are on an entity teaching task. Literature first analyzes the meaning expressed in books and then searches for the core words of the text based on artificial intelligence technology. This method can search a large number of real corpora and provide a wide range of reading resources for students. At the same time, university teachers can also construct different teaching activities from the corpus structure, which makes it more convenient to carry out student-centered task-based and inquiry teaching activities, and better exercise students' critical thinking, cross-cultural communication ability, as well as innovative thinking. This model breaks through the most traditional “classroom + textbook” teaching situation in the past, achieves student-centered task-based exploratory teaching, nurtures new interdisciplinary engineering talents deficient in new era emerging industries and new economies with new era technology, and promotes the development and progress of college English teachers' teaching to a certain extent.

RETRACTED

## 2. Related Work

### 2.1. AI and Education

AI has a history of more than 60 years since the Dartmouth conference put forward the concept of AI and became a discipline in 1956. AI and education is a cutting-edge interdisciplinary science involving computer science, information science, education, psychology, linguistics, neuroscience, and philosophy [12]. At present, the primary task of the development of artificial intelligence technology is to develop an intelligent information processing theory. From the beginning to the end, artificial intelligence technology has been aimed at building a computing system with human intelligent behavior. AI focuses more on the use of artificial methods and electronic technology to simulate and expand human intelligence, to achieve machine intelligence to a certain extent. Since the twenty-first century, AI technologies have breached many challenging intractable problems by combining big data processing through algorithms and deep learning, such as natural language processing, perception, moving and manipulating objects, reasoning, speech recognition, and image recognition [13, 14]. As one of the core technologies that drive the progress of modern society, AI is widely applied to agriculture, industry, medical care, and other areas, and various industries are actively using AI to crack industry problems and explore new directions and channels for industry development, and education is no exception.

We deeply study the current trend and possibility of the combination of college English and AI technology in teaching reform. First, from the perspective of English teachers, we have a deep understanding of the combination and research direction of AI and education at home and abroad.

### 2.2. College English Literature Classroom Teaching Model

Teaching methods and modes are the key factors that determine the effectiveness of teaching and learning; they are the structural framework that incorporates the teaching content. At present, China's College English teaching generally adopts multimedia equipment to assist classroom teaching tasks. However, this kind of classroom teaching method only helps to improve students' English listening, and students' deep understanding of the content of the textbook is not good. The current teaching mode should be combined with the four training goals of “listening, speaking, reading, and writing” in modern college English teaching. This also has considerable limitations, which usually show that the main body of classroom teaching is the teacher. This limitation makes teachers not only responsible for teaching but also responsible for designing the development and final evaluation of English teaching activities. Affected by the enrollment system of colleges and universities in China, there are a large number of college students and too large classes at present. Generally, it is difficult for teachers to get familiar with the actual situation of each student in a short time. Everyone's language ability practice takes time to accumulate, which leads to teachers' lack of objective understanding and evaluation of each student's actual learning situation at the English level, which will eventually reduce the overall quality of English teaching [15]..

RETRACTED

With the rapid development of AI in today's era, AI technology has been integrated into college English in educational reform. Therefore, the reasonable establishment of an intelligent classroom teaching system can deepen students' understanding and change the role of teachers. It can better express the emotion carried by English words and phrases in English literature class. This enables each student to quickly understand the main idea of each work in a more complex context, master the key points of English learning, and help students improve their basic reading ability and deep English subject quality. Therefore, it is worth thinking about how to realize AI technology.

## 3. Scheme or Model Design

The proposed model for analyzing the effect of reforming English literature classroom teaching on the theme of environmental protection in colleges and universities is shown in Figure 1. Firstly, we input the effect analysis index data, and the effect analysis index mainly consists of six aspects: teaching attitude, teaching methods, reform program, reformed teaching content, classroom organization, and teaching methods; then, we analyze the index data layer by layer using rank sum operation and hierarchical analysis method. Finally, we design the effect analysis model of English literature classroom teaching reform on the theme of environmental protection in colleges and universities given BP neural network, and by analyzing the data layer by layer, we establish three hidden layer neurons to fit the data and get the final effect analysis prediction results.

### 3.1. Rank Sum Operation

The rank sum operation is a method that uses the characteristic that rank can quantitatively analyze qualitative problems and synthesizes the ranking of all judges for the importance of all indicators, which can finally determine the weight of the indicator system conveniently and effectively. Several indicators were set, and different categories of people (teachers, classmates, etc.) were called to rate the reform of English literature classroom teaching on the topic of environmental protection. The importance serial number given by each expert is the expert's rank, and the rank sum is obtained by counting all the experts' ratings of the indicators, and the rank sum weight is determined as shown in the following equation:

(1) $$\begin{array}{c} w_{i}=\frac{2\left[s\left(1+m\right)-A_{i}\right]}{ms\left(1+m\right)}. \end{array}$$

Among them, *m* is the number of indicators, *s* is the number of experts, *A_i_* is the ranking sum of the *i*-th indicator by experts, and *w_i_* is the weight of the *i*-th indicator.

RETRACTED

In this paper, we use *x*^2^ to test whether the experts are consistent concerning the weights of the indicators, and the conformance test passes. Finally, the effect of teaching reform is analyzed. If the conformance test fails, you need to consult the expert again for a second calibration. The calculation of the conformance test is shown in the following equation:

(2) $$\begin{array}{c} x^{2}=\frac{m\left(s-1\right)S}{{\left(12\right)}^{-1}m^{2}\left(s^{3}-s\right)}, \end{array}$$

Among them, *S* = (*s*_1_^2^ + *s*_2_^2^+⋯+*s*_*n*_^2^) − ((*s*_1_ + *s*_2_+⋯+*s*_*n*_)/*n*).

### 3.2. Analytic Hierarchy Process

Analytic hierarchy process (AHP) refers to the process of complex and multicriteria decision-making problems as a system [16], decomposes the goals of solving the problem to obtain multiple small goals, and then decomposes the small goals into different subgoals at different levels. In the fuzzy quantitative method based on qualitative indicators, we calculate the hierarchical individual ranking and total ranking, and then calculate in sequence: According to the analytic hierarchy process, we decide the overall goal, sub-goals at all levels, evaluation criteria at all levels, and the order of the final specific plan. A relatively large decision-making problem is subdivided into different small hierarchical structures, and then, with the help of the eigenvector obtained by solving the judgment matrix, the weight of each level element relative to the upper-level element is calculated. Finally, the weighted summation algorithm is used to recursively calculate the final weight of each small-level scheme to the overall goal and determine the sub-scheme with the largest final weight result as the optimal scheme. The scheme with the highest weight is the best. The analytic hierarchy process is more suitable for decision-making problems where evaluation indicators are layered and staggered, and it is difficult to quantitatively describe the target value [17].

RETRACTED

The analytic hierarchy process for the sake of resolving the objectives to be achieved into several determines the constituent factors according to the nature of the research problem, hierarchizes the factors according to their interrelationship, forms a hierarchical model and analyzes them layer by layer, and finally determines the total weight of the indicator layer for the objective layer. First, a judgment matrix needs to be established, and the calculation formula is established as shown in the following equation:

(3) $$\begin{array}{c} J=\left\{\begin{array}{cccc} a_{1}=1 & a_{2}=\frac{w_{1}}{w_{2}} & \cdots & a_{1n}=\frac{w_{1}}{w_{n}}\\ a_{2}=\frac{w_{2}}{w_{1}} & a_{2}=1 & \cdots & a_{2n}=\frac{w_{2}}{w_{n}}\\ \cdot & \cdot & \; & \cdot \\ \cdot & \cdot & \; & \cdot \\ a_{n1}=\frac{w_{n}}{w_{1}} & a_{n2}=\frac{w_{n}}{w_{2}} & \cdots & a_{n}=1 \end{array}\right\}. \end{array}$$

Based on the relevant data, we establish the judgment matrix shown in Equation (3) to choose a more stable 9 scalar assignment method; the assignment standard of this method is shown in Table 1.

Firstly, a judgment matrix is established for each expert, then a weighted calculation is performed to solve the judgment matrix of the weights, and finally, the weights *w* = {*w*_1_, *w*_2_, ⋯, *w*_*n*_} of each layer of indicators are calculated separately, and the sum method is calculated as shown in Equation (4), and the root method is calculated as shown in Equation (5):

(4) $$\begin{array}{c} w_{i}=\frac{1}{n}\overset{n}{\underset{j=1}{\sum }}\frac{a_{j}}{\sum_{i=1}^{n}a_{j}}, \end{array}$$

(5) $$\begin{array}{c} w_{i}={\left(\overset{n}{\underset{j=1}{\prod }}a_{j}\right)}^{1/n}/\overset{n}{\underset{i=1}{\sum }}{\left(\overset{n}{\underset{j=1}{\prod }}a_{j}\right)}^{1/n}. \end{array}$$

### 3.3. BP Neural Network Modeling

Artificial neural networks are nonlinear, input and output mapping, flexible information processing systems composed of a great number of interconnected units that mimic neurons in the brain [18]. According to the differences in network structure and learning algorithms, artificial neural networks are classified into five categories: single-layer forward networks, multilayer forward networks, feedback networks, random neural networks, and competitive neural networks. Single-layer neural networks can only solve linear classification problems, multilayer neural networks can be used for nonlinear classification questions, and BP neural networks are the result of multilayer neural network learning algorithm training form [19, 20]. The BP network includes the forward transmission, the reverse transmission of the information, and the reverse transmission of the calculation error. It was a multilayer feed-forward network trained by the reverse transmission of errors. A typical BP network has three layers: the input, hidden, and output layers.

RETRACTED

The basic operation idea of the BP neural network is as follows: apiece nerve cell of the input layer was in charge of receiving the designated data samples and transferring them to each nerve cell of the hidden layer, and the neuron structure is demonstrated in Figure 2; the hidden layer carries out internal information processing and transformation according to the setting, which can be constructed as a single hidden node or multiple hidden layer structure, and the last hidden node can realize the transmission to the neural cells of the output network layer; after deeper information processing, the process of forwarding propagation is ended once, and finally, the output layer outputs the result. However, when the prediction result output by the network structure does not meet the error rate preset by the overall model, it will enter the error backpropagation stage. At this time, the error is back propagated to the implied layer and the input layer by using the improved algorithm of the BP neural network-gradient descent method to continuously correct the weight and threshold value of each layer. The two processes of forwarding propagation [21] and error back propagation [22, 23] are repeatedly alternated until convergence is reached; then, it is during the process of the BP intelligence network learning and training. The forward propagation calculation process is shown in Equations (6)–(7), and Equations (10)–(12) show the error backpropagation calculation process:

(6) $$\begin{array}{c} z=w_{0}x_{0}+w_{1}x_{1}+\cdots +w_{n}x_{n}, \end{array}$$

(7) $$\begin{array}{c} y=f\sum \begin{array}{c} n\\ i=0 \end{array}w_{i}x_{i}. \end{array}$$

It can be expressed in vector form, as shown in the following equations:

(8) $$\begin{array}{c} z=\sum \begin{array}{c} n\\ i=0 \end{array}w_{i}x_{i}=w^{T}x, \end{array}$$

(9) $$\begin{array}{c} y=f\left(w^{T}x\right), \end{array}$$

(10) $$\begin{array}{c} \Delta W=-\eta E^{`}, \end{array}$$

(11) $$\begin{array}{c} \frac{\delta E}{\delta W}=\frac{\delta \left(1/2\right){\left[t-f\left(w^{T}x\right)\right]}^{2}}{\delta w}, \end{array}$$

(12) $$\begin{array}{c} \Delta W=-\eta E^{`}=\eta \left(t-y\right)f^{`}\left(w^{T}x\right)x=\eta \delta x, \end{array}$$

where*δ* = (*t* − *y*)*f*^`^(*w*^*T*^*x*).

BP neural network is a supervised learning [24]. This paper adopts python as the programming language and uses the PyTorch deep learning framework developed by Facebook to establish BP neural network fitting scores to realize the analysis of the effect of English literature classroom teaching reform under the theme of environmental protection in universities.

RETRACTED

The network model for analyzing the effect of the English literature classroom teaching reform we proposed is shown in Figure 1. First, the rank sum operation and hierarchical analysis are performed on the survey scores to verify the consistency of the index weights; then, the qualified data are used as the input of the analysis model. The amount of the input layer's node depended on the size of the input measurement. We collect data by issuing questionnaires. A total of 300 copies were released, and 247 copies were effectively recovered. Through data processing, 200 of them are finally used. The scoring data are shown in Table 2. Finally, a BP neural network was used to model and analyze the effect of English literature classroom teaching reform for the theme of environmental protection in most colleges and universities, and the output layer node was set to 1 because of the final teaching reform affect analysis results.

For the survey about classroom reform, the statistics were visualized and analyzed as shown in Figure 3. Each survey indicator was formed into a dotted line graph to observe its fluctuation trend and analyze the fluctuation of the indicator under the reform of English literature classroom teaching on the theme of environmental protection in universities.

Neural networks generally contain one or more hidden layer nodes, and several studies have shown that a single hidden layer neural network can achieve nonlinear mapping by increasing the number of neurons; for more complex data, the number of hidden layers can be increased to linear partitioning and can be better performed by abstracting the features of input data into another dimension space and displaying its more abstract features. Therefore, when designing the model structure, this paper sets the number of hidden layers to 1, 2, and 3 for experiments and finally takes the group with the best fitting effect as the number of hidden layers. The number of neuron nodes in the hidden layer also has a significant impact on the final result of the whole network model, and the number of node neurons belongs to the empirical value. If the empirical value is too large, the model training time will be too long, and too small will lead to poor model results. In this paper, the number of hidden layer nodes is obtained by the empirical value calculation formula; the specific calculation is shown in the following equation:

(13) $$\begin{array}{c} H_{n}=\sqrt{m+l}+a\;1\leq a\leq 10. \end{array}$$

Among them, *H*_*n*_ is the number of neuron cells in the hidden layer, and *m* and *l* are the number of neurons in the input and output layers.

RETRACTED

## 4. Experimental Analysis

### 4.1. Experimental Environment

For sake of better validating our suggested model of teaching effect analysis of English literature classroom reform on the theme of environmental protection in colleges and universities, multiple data obtained through the survey were saved as self-built datasets after data preprocessing.  Table 3 shows the software environment used for model training in this paper, and Table 4 lists some hardware experimental environments.

### 4.2. Model Learning Process

The model structure based on BP neural network has three layers, which have the characteristics of multiple inputs, one output, and multiple neuron nodes in the hidden layer. In general, the gradient descent algorithm adjusts and modifies the connection weight of the network through the backpropagation of the output error at each step of the network structure; after multiple back-propagation derivations, the error is minimized. The whole learning process is shown in Figure 4.

Firstly, the parameters are initialized for the analysis model of the effect of reforming English literature classroom teaching on the theme of environmental protection in colleges and universities, and the basic model structure is established. Then, a sample of the survey data is entered into the model, the number of hidden layer neuronal nodes in the network is calculated from the input data, and the final fitted data is exported through the cooperation of multiple neurons. The global sum of squares error of the model structure is calculated for the obtained response value, and the error is used to determine whether the model prediction is completed. If the error is large, continue to calculate the inverse error, recalculate the number of nodes in the hidden layer, output the response value, and recalculate the global sum of squares error of the model. When the minimum error tends to be flat and no longer changes, the weight information is the final model weight.

### 4.3. Experimental Results Analysis

The loss results of the model training process in this paper are shown in Figure 5. The model loss calculation method adopts the mean square error function, and the calculation result is shown in Equation (14). It can be seen from the figure that the analysis model of environmental protection teaching reform in College English literature classrooms is close to fitting after about 15 rounds of training, and the final simulation error is about 0.0192.

(14) $$\begin{array}{c} MSE\left(y,y^{`}\right)=\frac{\sum \begin{array}{c} n\\ i=1 \end{array}{\left(y-y^{`}\right)}^{2}}{n}. \end{array}$$

Different model structures also have a great impact on the final analysis effect of the model. We not only need to train data to get the optimal model based on data but also get the current optimal analysis model by analyzing the network model under different structures and parameters.

RETRACTED

BP neural network can contain one or more hidden layers, and related research shows that by increasing the number of neurons, the single-layer BP network can map all continuous functions. Therefore, in this paper, three different hidden layer neural network structures are designed to fit the model, and the training loss of a different number of hidden layers is shown in Figure 6.

The final model was tested and analyzed for three times, and the final analysis on the effect of classroom teaching reform of English literature on the theme of environmental protection in colleges and universities was obtained. The results are shown in Table 5. Using the trained model weight parameters, we made three predictions in the three-layer hidden layer model, and the results are shown in the first three rows in the table. We averaged all the final test results, as shown in the last row of the table. According to the data shown in the table, we can see that the current reform of English literature teaching has brought remarkable results to AI technology, and the students and teachers are both more agreeable to the teaching model and have higher ratings.  Figure 7 shows the results of model analysis of the effect of English literature teaching reform with the theme of environmental protection in colleges and universities.

From the results of the visualization, the results of multiple tests are stable, indicating that the model is in a stable state. For each different index, it can be roughly seen that the reform of combining AI technology with English literature classroom teaching on environmental protection topics in colleges and universities has achieved good results and the model analysis scores are all above 80 points. The point cloud visualization of the results of the reformed teaching content in the classroom of English literature theme of environmental protection in colleges and universities with AI technology in Table 2 is shown in Figure 8, which shows that the reformed teaching content has a relatively high score, mostly given 90 or more, while the reform reasonability is in the reformed teaching content item is relatively high, mostly given 90 or above, while the reform reasonability item is in the middle, mostly around 85. This is also consistent with the predictions of the model presented in this paper.

RETRACTED

## 5. Conclusions

Because of the teaching effect analysis of the classroom teaching reform of English literature on the theme of environmental protection in colleges and universities, this paper uses the analytic hierarchy process and BP neural network to propose a classroom teaching evaluation model and applies it to the field of analyzing the effect of the current university teaching reform. First, set up several effect analysis indicators, and establish the analysis and investigation database of teaching reform through campus investigation. Secondly, rank sum operation and analytic hierarchy process are used to preprocess the data based on expert scoring. However, when the prediction result output by the network structure does not meet the error rate preset by the overall model, the model will enter the back propagation stage again and recalculate the error rate and weight parameters. Through the survey data fitting model, the final analysis results of classroom teaching reform effect of English literature on environmental protection in colleges and universities based on AI technology are obtained.

The scores of the model based on the BP neural network under the six effect analysis indicators of teaching attitude, teaching tools, reform plan, reform teaching content, classroom organization, and reform rationality are 90.97, 86.3, 80.4, 95.7, 84.8, and 87.4, respectively. It can be seen from the results that the model can effectively analyze the situation of classroom reform and improve the time and accuracy of the current teaching reform analysis, which has a certain practical application value.

## Figures and Tables

**Figure 1:** A model for analyzing the effect of reforming English literature classroom teaching on the theme of environmental protection in colleges and universities.

**Figure 2:** Neuronal structure.

**Figure 3:** Trend of fluctuation of survey results.

**Figure 4:** Analysis of model structure learning process.

**Figure 5:** Loss curve.

**Figure 6:** Different hidden layer loss curves.

**Figure 7:** Visualization of model analysis results.

**Figure 8:** Point cloud visualization of survey results.

**Table 1:** Scale assignment criteria.

Scale (*w*_*i*_/*w*_*j*_)	Meaning
1	Indicates the influence factor *v_i_* is equally important as compared to *v_j_*, *v_i_* is equally important as compared to *v_j_*
3	Indicates that the influence factor *v*_i_ is slightly more important than *v_j_*, *v_i_* than *v_j_*
5	Indicates that the influence factor *v_i_* is significantly more important than *v_j_*
7	Indicates that the influence factor *v_i_* is significantly more important than *v_j_*
9	Indicates that the influence factor *v_i_* is significantly more important than *v_j_*
2, 4, 6, 8	The median

RETRACTED

**Table 2:** Survey on the effect of reforming English literature teaching on the theme of environmental protection in universities.

Investigator number	Teaching attitude	Teaching tools	Reform program	Reformed teaching content	Classroom organization	Reform reasonableness
1	92.5	87.6	98	97	82	87.3
2	91	89.5	92	90.9	85.4	85
3	94	82.9	88.7	96.3	90.5	89
…	…	…	…	…	…	…
198	87.2	91.3	82	85.7	91.6	82.1
199	93.5	86	91.4	90	97	91
200	89	96	99	79	70.5	92.4

**Table 3:** Experimental software environment.

Environment	Description
Python	Development languages
PyTorch1.7	Deep learning framework
Nvidia CUDA 10.1	Deep learning acceleration library
CuDNN-V7.6	Deep learning acceleration library

**Table 4:** Experimental hardware environment.

Environment	Description
Windows 10	Operating system
32G	CPU memory size
Nvidia Tesla T4	Deep learning dedicated graphics card
1 T	SSD
Intel Core i7 @2.30 Hz	CPU

**Table 5:** Results of the model analysis of the effect of reforming English literature teaching on the theme of environmental protection in universities.

Test NO	Teaching attitude	Teaching methods	Reform programs	Reformed teaching content	Classroom organizational	Reform reasonability
1	89	85	90	95	80	88
2	92.1	87.8	90.3	96.7	84.8	86.4
3	91.8	86.1	91	95.5	89.5	87.9
Average	90.9	86.3	90.4	95.7	84.8	87.4

## Data Availability

The dataset can be accessed upon request.
